# Effects of Qigong Therapy on the Anaerobic Threshold in Patients with Stable Coronary Artery Disease: A Randomized Controlled Trial

**DOI:** 10.1155/2022/5690569

**Published:** 2022-09-14

**Authors:** Fengrun Zhao, Chen Liang, Christopher John Zaslawski, Zhenyu Cao

**Affiliations:** ^1^College of Acupuncture and Massage, Nanjing University of Chinese Medicine, Nanjing 210023, Jiangsu, China; ^2^Institute of Sports Medicine, General Administration of Sport of China, Beijing 100061, China; ^3^University of Technology, Sydney 2007, Australia

## Abstract

**Objective:**

This study aims to identify whether Qigong (QG) rehabilitation therapy can significantly improve the cardiac function of patients with stable coronary artery disease (SCAD) compared with routine therapy. Thus, a randomized controlled trial was conducted to evaluate the curative effects of a three-month QG rehabilitation therapy on cardiac rehabilitation. *Patients and Methods.* In this trial, a total of 68 patients with SCAD were randomly divided into the QG group (34 patients) and the control (CON) group (34 patients). Patients in the CON group received routine cardiologic medication without any special intervention. Based on the treatment in the CON group, patients in the QG group were provided additionally with a 12-week traditional Chinese medicine (TCM) cardiac rehabilitation QG exercise training program. The outcomes of these patients were assessed at baseline and after 12 weeks of intervention through the treadmill (anaerobic threshold (AT)) test.

**Results:**

After 12 weeks of intervention, the AT, volume of oxygen (VO2), oxygen uptake/kilogram (VO2/kg), metabolic equivalents (METS), and oxygen pulse (VO2/HR) of patients in the QG group were significantly higher than those of patients in the CON group (*P* < 0.05).

**Conclusion:**

QG therapy can achieve certain curative effects and safety for patients with SCAD. This trial is registered with *Clinicaltrials*.*gov identifier* (ChiCTR1800015823).

## 1. Introduction

Exercise training intervention can reduce the overall mortality of patients with heart diseases. Monitored exercise training is also an important component of a comprehensive cardiac rehabilitation plan [1, 2]. The potential cardioprotective effect of regular sports has been confirmed by clinical evidence, which shows that long-term regular aerobic endurance training can increase the risk factors of cardiovascular diseases [3]. The QG therapy training is similar to the aerobic training, but it has some distinct characteristics. For instance, it can regulate the body, breathing, and psychology of individuals who conduct this training program [4]. QG exercise prescription refers to that rehabilitation where doctors or physiotherapists prescribe the type, intensity, time, and frequency of QG exercise in the form of prescription, put forward matters needing attention in the QG exercise, and make patients achieve rehabilitation through regular training. However, there is not enough evidence to support the effectiveness and safety of QG therapy in cardiac rehabilitation.

The anaerobic threshold (AT) refers to the level of oxygen uptake during exercise in a cardiopulmonary exercise test. Beyond this level, anaerobic metabolism will supplement aerobic metabolism to produce energy. The higher the AT is, the stronger the aerobic function is. According to previous studies, moderate-intensity aerobic exercise training can improve the AT of patients with heart diseases, which provides a strong basis for the formulation of clinical cardiac rehabilitation exercise treatment plans [5]. However, there is no relevant research on the improvement of AT in patients with heart disease through QG therapy training. In order to identify whether QG therapy training can improve the AT of patients with heart diseases, a randomized trial was conducted to compare two strategies by evaluating the indexes related to the AT in a cardiopulmonary exercise treadmill test. These findings may provide a basis for clinicians to formulate standardized QG therapy exercise prescriptions.

## 2. Methodology

### 2.1. Ethical Approval

In this study, all procedures involving human participants were performed under the Declaration of Helsinki (1964), relevant amendments, and regulations for Chinese clinical trials. The Ethics Committee of Sports Medicine Hospital Affiliated to General Administration of Sport of China reviewed and approved the protocol (2017020). All participants signed written informed consent before enrollment.

### 2.2. Trial Design

In this randomized controlled trial, all patients were divided into the QG group and the CON group with a random number table. All participants met the consecutive inclusion criteria. The program was registered in the China Clinical Trial Registry (ChiCTR1800015823).

### 2.3. Design

In this study, a total of 68 patients with SCAD who were treated in the Functional Testing Department of the General Administration of Sport of China Sports Medical Science Institute from March 2017 to September 2017 were included and randomly divided into the cardiac rehabilitation QG group (*n* = 34) and the CON group (*n* = 34). In the QG group, 4 patients quit the study due to failure to complete the whole training program, and the remaining 30 patients completed the 12-week training program. In the CON group, 5 patients were excluded due to failed connection of their phones. Eventually, a total of 29 participants completed the study (Figure 1).

The diagnostic criteria for SCAD are presented as follows: (i) a reversible supply/demand mismatch related to ischemia, a history of myocardial infarction; (ii) stable, usually asymptomatic, disease at different stages after acute coronary syndrome; and (iii) long-term, quiescent, and presymptomatic state of coronary atherosclerosis. Anyone who can satisfy the above criteria can be diagnosed as having SCAD [6]. In the study, the inclusion criteria included (i) patients who satisfied the diagnostic criteria of SCAD; (ii) patients who were discharged from the hospital 2–3 or more months; (iii) patients who were assessed to be the New York Heart Association functional classification I–III; (iv) patients who aged 40–70 years; (v) patients who had an education background of junior high school or above; (vi) patients who had no exercise intervention in the previous month; (vii) patients who may be accompanied by hypertension, diabetes, dyslipidemia, cerebrovascular disease, smoking, drinking, sleep disorders, and psychological stress; (viii) patients who received artery bypass, coronary intervention, or no surgery; and (ix) patients who administered cardiovascular drugs, such as aspirin, clopidogrel, angiotensin-converting enzyme inhibitors (ACEI), angiotensin II receptor blocker (ARB), calcium channel blockers (CCB), diuretic, statins, oral hypoglycemic agent, and insulin. The exclusion criteria included (i) patients with uncontrolled tachycardia (heart rate (HR) > 120 beats/min); (ii) patients with uncontrolled shortness of breath (quiescent frequency >30 beats/min); (iii) patients with uncontrolled respiratory failure (blood oxygen saturation ≤90%); (v) patients with uncontrolled hypertension (systolic blood pressure (BP) >180mm·Hg or diastolic BP > 110mm·Hg in the preexercise assessment); (v) patients with changes in the body weight ± 1.8 kg before 72 h; (vi) patients with uncontrolled high glucose (random blood glucose >18 mmol/l); (vii) patients with uncontrolled malignant arrhythmia that could cause hemodynamic instability; (viii) patients who were diagnosed or suspected to have pseudoaneurysm or preoperative arterial dissection; (ix) patients with uncontrolled septic shock and sepsis; (x) patients with severe valvular disease before surgery or cardiac heart disease in the acute phase of heart failure; (xi) patients who may develop aggravated diseases in the nervous or motor system or rheumatic disease due to exercises; (xii) patients who had poor compliance (Table 1).

Those participants who voluntarily withdrew from this trial due to objective or subjective reasons, had failure to complete the training program or had incomplete cardiopulmonary exercise test data were excluded from the final analysis.

### 2.4. Intervention and Methods

Patients in the CON group received routine cardiologic medication without any special intervention. Based on the treatment in the CON group, patients in the QG group were provided additionally with a 12-week TCM cardiac rehabilitation QG exercise training program (3–6 sets of exercises each time for 40–60 min in total, 6–7 times a week). The training was guided by a sports medicine exercise prescription research team from a national institute. These patients completed the training program collectively in the Beijing gymnasium supervised by two doctors from our team. After completing the training program, they were asked to fill out the sports record form delivered by our team members.

In this study, the cardiac rehabilitation QG exercise involved upper extremities, lower extremities, breathing, self-massage, and even the whole body. These moderate-intensity exercises were in line with the principles of modern exercise physiology. Besides the preparation and ending postures (leading qi to its origin), the whole set of exercises also included other eight postures, namely, Lotus Nirvana posture, cardiac protection posture, respiratory opening and closing posture, heart channel massage posture, Taiji single whip posture, left-right glance posture, left and right turning posture, and wild goose flying posture (Figure 2). Patients completed these postures in a sequence. With the consideration of modern sports rehabilitation, the training program was designed to improve cardiopulmonary function, muscle strength, flexibility, and balance.

### 2.5. The CON Group

Patients in the CON group did not undergo any exercise intervention.

### 2.6. Quality Control

The training program was completed within 13 weeks. In the first week, patients in the QG group were guided to conduct exercises by qualified instructors for 40 min/day. At the end of the week, the researchers determined that the patient was able to complete the full set of actions accurately after a unified assessment. Then, the patients began to conduct the 12-week training program. For home exercises, patients shall upload the training records to the WeChat group every day. All patients were required to complete exercises during the period, including the collective training three times a week.

### 2.7. Collection of Primary End Points and Secondary End Points

#### 2.7.1. Primary End Points

Cardiopulmonary exercise test: in the cardiopulmonary exercise test (CPET), the respiratory gas monitoring technology (COSMED Quark PFT ergo; COSMED offices, Rome, Italia), the Shuntai Tango + Tablet sports BP monitor (activity tablet; SunTech Medicial, Morrisville, USA), or treadmill (h/p/cosmos) technology (h/p/cosmos, Munich, Germany) were adopted to detect the dynamic changes of CPET parameters and carbon dioxide emission under different load conditions in real time. The modified Bruce protocol was utilized to perform the graded CPET. The heart rate (HR) and BP of patients were collected at the last minute of each level of exercises. The rating of perceived exertion and the changes in the ST segment of the electrocardiogram (ECG) were recorded.

### 2.8. Follow-Up

Twelve weeks after the intervention, the CPET parameters of these patients were collected. In the QG group, 4 patients could not complete the training program and quit the trial. In the CON group, 5 patients quit the trial due to failed connection. Other patients completed the CPET.

### 2.9. Safety Assessment

The termination criteria of the exercise arterial were established based on the guidelines of the American College of Sports Medicine. This trial was terminated when the following symptoms occurred, including abnormal ECG or high BP; maximum HR or heart failure; typical chest pain and chest tightness; difficulty in breathing; and ECG ST-T segment reduction and reactive hypotension.

### 2.10. Sample Size and Statistical Method

According to previous studies, the exercise training intervention increased the peak VO2/kg in the primary endpoint index by 30%. Through the calculation based on the sample size formula, 29 SCAD patients at the rehabilitation stage III (90% power; 5% significance level; and two-sidedlog-rank test) were obtained from each group. There were 58 patients in total in the two groups. The final estimated sample size would include 64 patients after adding 10% of the withdrawal patients (about 6 patients), namely, 32 patients in each group.

The count data were expressed as a percentage. The normally distributed data among the measurement data were expressed as mean ± SD. Data were statistically analyzed with SPSS 20.0 (International Business Machines, Armonk, New York, USA). The normality of the data distribution was evaluated based on the Kolmogorov–Smirnov test results. A significant difference was made with the analysis of covariance and Fisher's least significant difference test. *P* < 0.05 indicated that there was a significant difference.

## 3. Results

### 3.1. Demographic Characteristics

There was no significant difference in the demographic characteristics of these patients, including gender, age, duration of disease, height, weight, body mass index (BMI), surgical history, complications, and cardiovascular disease (CVD) medication (*P* > 0.05; Table2). The administration of therapeutic drugs did not change during intervention.

### 3.2. Analysis of Anaerobic Threshold Parameters in a Cardiopulmonary Exercise Test

After 12 weeks of intervention, VO2, VO2/kg, METS, and VO2/HR of patients in the QG group were significantly higher than those of patients in the CON group (*P* < 0.05; Table 3).

There was no significant change in time, speed, grade, HR, stroke volume (SV), ventilation volume/oxygen uptake (VE/VO2), and ventilation over carbon dioxide elimination (VE/VCO2) between the two groups (*P* > 0.05; Table 3).

### 3.3. Safety Assessment

No adverse events occurred in patients in both the groups.

## 4. Discussion

In this study, the results demonstrated that QG can improve the AT and CPET parameters of SCAD patients who received rehabilitation treatment.

As per previous studies, QG therapy training is considered safe and effective in the treatment of CVD patients [7–11]. As a guiding intensity of exercise, anaerobic threshold intensity can scientifically and effectively guide the formulation of aerobic exercise prescriptions [12]. Exercise therapy based on AT exercise schemes can ensure the safety of exercises from the perspective of hemodynamics. Specifically, it can effectively improve the level of oxygen metabolism and exercise tolerance, improve the abnormal exercise response of patients, and prevent the occurrence of malignant cardiovascular events during exercises [13–15].

The results of this study revealed that several important parameters (such as VO2, VO2/kg, metabolic equivalent, VO2/HR, stroke output, and cardiopulmonary aerobic exercise response ability) of patients in the QG group at the AT level were significantly improved compared with the CON group. It indicated that QG therapy training could improve the aerobic ability, cardiovascular efficiency, and cardiac pumping ability of patients. Increasing cardiopulmonary exercise tolerance at the AT level in patients with cardiovascular diseases can effectively delay the progression of diseases and improve the prognosis of patients. The mechanism may be related to the “uniform, thin, and uniform and long” thoracoabdominal combined breathing method, which contributed to the balance of the autonomic nervous system, thus decreasing the abnormal excitation of sympathetic nerves and reducing blood pressure [16, 17]. Besides, it may also correlate with the formation of cardiac collateral circulation, the improvement of coronary blood supply, and the improvement of myocardial contractility [18, 19]. In addition, this mechanism may be associated with the enhanced oxygen uptake capacity of skeletal muscles, increased arterial and venous oxygen difference, decreased blood supply of peripheral muscle metabolism, and reduced cardiac load and myocardial oxygen consumption. Furthermore, it may also be affected by the enhanced muscle oxygen utilization capacity and metabolic capacity, which can improve cardiovascular efficiency, significantly enhance patients' exercise endurance and maximum oxygen consumption, and reduce fatigue [20–22]. The QG therapy can improve the muscle adaptability of patients. In QG therapy, the CON force of lower limbs can be enhanced through the practice of squatting pile, horse step, bow step and virtual step, and the alternating stress of both lower limbs during practice. At the same time, this rhythmic stimulation could increase the density and number of muscle capillaries of the lower limbs. That is to say, the opening number and diameter of capillaries become larger, which can relatively improve the diffusion area and efficiency of the blood cell gas exchange during muscle exercises. The enhanced oxygen uptake capacity of the skeletal muscles will increase the arteriovenous oxygen difference, reduce the blood supply of peripheral muscle metabolism, and finally reduce the cardiac load and myocardial oxygen consumption.

These findings suggested that the improvement of various indexes related to the AT in SCAD patients by QG may be related to a variety of mechanisms. QG therapy training reflects the full combination of aerobic training, resistance training, and stretching exercises. This therapy can produce cardiac protective effects by mitigating atherosclerosis, psychological disorders, thrombosis, ischemia, and arrhythmia. Based on that, it can improve the resistance of cardiovascular and skeletal muscles, strengthen exercises, generate a good mood, and finally reduce the mortality of cardiovascular diseases [7, 23, 24].

According to the results of this study, this cardiac rehabilitation QG therapy is effective and safe for SCAD patients at the rehabilitation stage III. In addition, it is easy to implement this therapy, which can be accepted by patients with SCAD. Moreover, it can provide an effective intervention means for the lifelong rehabilitation of these patients. However, there are still many points to be explored in the research on the intervention of TCM in modern cardiac rehabilitation. It is necessary to further explore the cardiac rehabilitation QG therapy and perform an analysis of it in terms of exercise intensity, exercise frequency, exercise time, action standardization, quantification, and improvement effect mechanism.

At the same time, the focus of this study is only placed on patients with SCAD. Therefore, different QG training programs can be provided for patients with other disease types(such as heart failure, post percutaneous coronary intervention (PCI), and arrhythmia) and various rehabilitation stages (such as acute stage and inpatient stage (stage I and II)). Similarly, it is also necessary to take account of stratification factors in subsequent studies, including gender, course of disease, and medication. The QG exercise schemes with different intensities, different time lengths, and different frequencies can be designed for different patients in order to achieve favorable outcomes. QG is rooted in ancient Chinese philosophy. Hence, it is also required to combine the profound TCM QG theory with modern medical knowledge to scientifically explain relevant mechanisms in subsequent studies.

These findings of this study provide an effective method and theoretical basis for the rehabilitation of SCAD patients within the AT. Nevertheless, there are still some limitations in this study, including the small sample size, short intervention cycle, and failure to evaluate the long-term effect of this training program. In addition, the experimental results need to be verified by repeated experiments. Although QG therapy has achieved some curative effects in patients with SCAD, it is also a demand to expand the sample size and improve the intervention methods for further validation research.

## 5. Conclusion

Through this study, it can be proved that QG therapy can achieve certain curative effects and safety in the rehabilitation treatment of patients with SCAD.

## Figures and Tables

**Figure 1:** Flow diagram of study subject recruitment.

**Figure 2:** Presentation of cardiac rehabilitation qigong exercise.

**Table 1:** Inclusion and exclusion criteria.

Inclusion criteria	(i) Meets the diagnostic criteria of SCAD; (ii) 2-3 or more months after discharge; (iii) the New York heart association functional classification I–III; (iv) those aged 40–70 years; (v) junior high school or above; (vi) no exercise intervention was taken in the previous month; (vii) patients may be accompanied by hypertension, diabetes, dyslipidemia, cerebrovascular disease, smoking, drinking, sleep disorders, and psychological stress; (viii) the patient has had artery bypass, coronary intervention, or no surgery; and (ix) cardiovascular drugs being taken include aspirin, clopidogrel, angiotension converting enzyme inhibitors (ACEI), angiotensin II receptor blocker (ARB), calcium channel blockers (CCB), diuretic, statins, oral hypoglycemic agent, insulin, or others.

Exclusion criteria	(i) Uncontrolled tachycardia (heart rate (HR) > 120 beats/min); (ii) uncontrolled shortness of breath(quiescent frequency >30 beats/min); (iii) uncontrolled respiratory failure (blood oxygen) saturation ≤90%; (v) uncontrolled hypertension(preexercise assessment systolic blood pressure (BP) >180 mm·Hg or diastolic BP > 110 mm·Hg); (v) change in body weight ± 1.8 kg before 72 h; (vi) uncontrolled high glucose (random blood glucose >18 mmol/l); (vii) uncontrolled malignant arrhythmia leading to hemodynamic instability; (viii) diagnosed or suspected pseudoaneurysm and preoperative arterial dissection; (ix) uncontrolled septic shock and sepsis; (x) severe valvular disease before surgery or cardiac heart disease in the acute phase of heart failure; (xi) exercise may lead to worsening the nervous system, motor system disease, or rheumatic disease; and (xii) patients cannot cooperate or are unwilling to cooperate.

**Table 2:** Changes of anaerobic threshold parameters in the cardiopulmonary exercise test in the QG training group, and the CON group.

	The QG group		The CON group		Z	*P*
	Baseline	Week 12	Baseline	Week 12		
Anaerobic threshold indicator appeared						
Time (min)	7.37 ± 3.71	7.75 ± 4.50	8.76 ± 3.84	8.62 ± 3.71	−0.762	>0.05
Speed (Kmh × 10)	34.93 ± 8.34	37.62 ± 10.79	36.79 ± 11.90	37.66 ± 10.04	−0.568	>0.05
Grade (%)	10.38 ± 2.73	11.09 ± 2.89	11.58 ± 1.92	11.38 ± 2.30	−0.20	>0.05
Anaerobic threshold response						
VO_2_ (ml/min)	1155.13 ± 432.89	1209.39 ± 461.46	1104.38 ± 488.03	1068.10 ± 292.02^#^	−2.12	<0.05
VO_2_/Kg (ml/min/kg)	16.77 ± 6.60	19.75 ± 6.40^*∗*^	17.10 ± 6.53	16.56 ± 4.45^#^	−2.27	<0.05
METS	4.8 ± 1.96	5.14 ± 1.82^*∗*^	4.86 ± 1.85	4.0 ± 1.54^#^	−2.19	<0.05
Anaerobic threshold cardiovascular response						
HR (bpm)	104.37 ± 18.44	106.57 ± 21.99	109.39 ± 20.31	108.38 ± 25.63	−0.335	>0.05
VO_2_/HR (ml/bpm)	9.97 ± 3.47	10.79 ± 3.35^*∗*^	9.76 ± 3.54	9.17 ± 2.25^#^	−2.47	<0.05
SV	69.70 ± 19.71	73.68 ± 21.04	67.48 ± 18.18	70.90 ± 24.41	−0.70	>0.05
Anaerobic threshold cardiovascular gas exchange						
VE/VO_2_	29.47 ± 4.63	29.93 ± 3.24	28.93 ± 3.54	28.45 ± 4.09	−1.55	>0.05
VE/VCO_2_	31.63 ± 5.68	31.39 ± 3.64	30.72 ± 4.25	29.93 ± 3.70	−1.47	>0.05

Data are expressed as mean ± SD. QG, qigong group; HR, heart rate; METS, metabolic equivalents; SV, stroke volume; VE/VCO_2_, ventilatory equivalents for carbon dioxide; VE/VO_2_, ventilatory equivalents for oxygen. ^*∗*^*P* < 0.05 versus^#^. ^#^The data in the table.

**Table 3:** Comparison of baseline demographic characteristics.

	Total	The QG group (*n* = 30)	The CON group (*n* = 29)	*P*
Sex (*n* (%))				
Male	17 (28.8)	10 (33.3)	7 (24.1)	0.436
Female	42 (71.2)	20 (66.7)	22 (75.9)	
Average age (mean ± SD) (y)	60.95 ± 5.15	61.23 ± 5.24	60.66 ± 5.85	0.843
Course of disease (mean ± SD) (y)	4.36 ± 2.02	4.73 ± 2.08	3.97 ± 1.92	0.147
Height (mean ± SD) (cm)	163.34 ± 6.89	163.5 ± 7.48	163.17 ± 6.34	0.857
Weight (mean ± SD) (kg)	63.86 ± 10.01	63.04 ± 10.53	64.71 ± 9.56	0.527
BMI (mean ± SD) (kg/m^2^)	23.81 ± 2.52	23.47 ± 2.47	24.17 ± 2.58	0.293
History of surgery (*n* (%))				
Coronary artery bypass	8 (13.6)	5 (16.7)	3 (10.3)	0.950
Coronary intervention	19 (32.2)	11 (36.7)	8 (27.6)	
No	32 (20.3)	14 (46.7)	18 (62.1)	
Combined disease (*n* (%))				
Hypertension	51 (86.4)	28 (93.3)	23 (79.3)	0.916
Diabetes	12 (20.3)	7 (23.3)	5 (17.2)	
Dyslipidemia	46 (78.0)	26 (86.7)	20 (69.0)	
Cerebrovascular disease	8 (13.6)	3 (10.0)	5 (17.2)	
Smoking	33 (56.0)	18 (60.0)	15 (51.7)	
Drinking	30 (50.8)	14 (46.7)	16 (55.2)	
Sleep disorder	38 (64.4)	17 (56.7)	21 (72.4)	
Psychological stress	21 (35.6)	11 (36.7)	10 (34.5)	
CVD drugs (*n* (%))				
Aspirin	47 (79.7)	26 (86.7)	21 (72.4)	0.936
Clopidogrel	18 (30.5)	10 (33.3)	8 (27.6)	
ACEI	33 (55.9)	17 (56.7)	16 (55.2)	
ARB	14 (23.7)	8 (26.7)	6 (20.7)	
CCB	18 (30.5)	10 (33.3)	8 (27.6)	
Diuretic	6 (10.2)	4 (13.3)	2 (6.9)	
Statins	35 (59.3)	15 (50.0)	20 (69.0)	
Oral hypoglycemic agent	2 (28.8)	2 (6.7)	0 (0)	
Insulin	3 (3.4)	2 (6.7)	1 (3.4)	
Others	19 (32.2)	10 (33.3)	9 (31.0)	

ACEI: angiotensin-converting enzyme inhibitor; ARB: angiotensin receptor blocker; CCB: calcium antagonist; CVD: cardio-vascular disease; QG: qigong group; CON: control group.

## Data Availability

The data that support the findings of this study are within the article, as well as available from the corresponding author upon request.
